The article "Measuring the Awareness of Chronic Kidney Disease (CKD) with Environmental Evaluation among Adult Diabetic Patients in Hail Region, Saudi Arabia" was retracted in 2023. Reasons: unreliable results or conclusions; concerns about the data; concerns about the peer review; concerns about the citations.

# Measuring the Awareness of Chronic Kidney Disease (CKD) with Environmental Evaluation among Adult Diabetic Patients in Hail Region, Saudi Arabia

**DOI:** 10.1155/2022/4505345

**Published:** 2022-06-29

**Authors:** Alreshidi Nahlah Fahad, Abdulrahman Ahmed Alkhateeb, Abdulrahman Rabah Alsharari, Abdulrhman Naif Alharbi, Alazmmy Abdullaziz Hamed

**Affiliations:** ^1^Assistant Professor, Endocrine Specialist, College of Medicine, University of Hail, Ha'il, Saudi Arabia; ^2^College of Medicine, University of Ha'il, Ha'il, Saudi Arabia

## Abstract

**Introduction:**

Chronic kidney disease (CKD) is one of the main chronic complications of T2DM that happens among T2DM patients who have uncontrolled glucose. Because CKD is considered a silent disease, the diagnosis is usually made at late stages when there will be few chances to prevent the adverse outcome.

**Aim:**

The goal of this study was to assess adult diabetic patients' awareness of developing chronic kidney disease at the community level in Hail region, Saudi Arabia, in 2022. *Patients and Methods*. This is a cross-sectional study conducted among diabetic patients in the Hail region, Saudi Arabia. A self-administered questionnaire translated into Arabic was distributed among patients with DM. The questionnaire covers social and demographic variables (such as age, gender, relationship status, and so on) as well as a 7-item questionnaire to assess the DM population's knowledge of CKD.

**Results:**

400 DM patients responded to our survey (51% females vs 49% males). Patients who were diagnosed with type 2 diabetes were 23.8% and 40.5% had a diabetes duration of 5–15 years. Nearly half (46.8%) were considered as a poor level of awareness, 29.3% had a moderate, and 24% had a good awareness level. Factors associated with an increased level of awareness were being a bachelor's degree, being unmarried, being a student, and having a doctor as a source of CKD information.

**Conclusion:**

There was a deficiency in the level of awareness among the diabetic patients in our region. Patients who were single with better education and who were well informed by the doctors about CKD information tend to be more aware of CKD as compared to other DM patients. Further research is warranted in order to establish the awareness level of DM patients regarding CKD and its complications.

## 1. Introduction

Diabetes mellitus (DM) is a collection of metabolic abnormalities defined by elevated blood glucose levels caused by a deficiency in circulating insulin, insulin resistance, or overproduction of hormones that inhibit insulin function [1]. From an epidemiological point, diabetes mellitus is one of the most common causes of death, disability, and economic loss worldwide. WHO predicted that by 2030, 366 million people will establish DM [2, 3]. Diabetes is classified into three types: type 1 (T1DM), type 2 (T2DM), and gestational diabetes. Type 1 DM mainly occurs secondary to an autoimmune destruction of beta cells in the islets of Langerhans in the pancreas, leading to a reduction in insulin secretion. T2DM occurs due to a defect in the action of insulin because of insulin resistance by body tissues [4]. Chronic complications are considered major consequences of T2DM which will impact the quality of life of patients. Chronic kidney disease (CKD) is one of the most common chronic consequences of T2DM in adults with uncontrolled glucose levels. [5] Diabetes is considered the leading cause of chronic kidney disease, 44% of CKD patients suffered from DM. Up to 77% of DM patients missed diagnosis with CKD. T2DM patients who have CKD are at risk for coronary artery disease as well [6, 7]. Because CKD is considered a silent disease, the diagnosis usually made at late stages, when there will be few chances to prevent the adverse outcome [8]. Loss of opportunities for prevention with insufficient care will lead to disease progression [9–14]. Because of lacking in the data that shows the awareness level regarding CKD among adult diabetic patients in the Hail region, Saudi Arabia, our aim in this study is to determine awareness and encourage it.

The article "Measuring the Awareness of Chronic Kidney Disease (CKD) with Environmental Evaluation among Adult Diabetic Patients in Hail Region, Saudi Arabia" was retracted in 2023. Reasons: unreliable results or conclusions; concerns about the data; concerns about the peer review; concerns about the citations.

## 2. Methods

This is a cross-sectional research conducted during 11 April to 18 May, 2022, among diabetic patients in the Hail region, Saudi Arabia. A self-administered questionnaire translated into Arabic was distributed among patients with DM. The Ethical Committee of the University of Hail's College of Medicine gave their approval prior to the start of the study initiation (approved number H-2022-190). With a 95 percent confidence interval and a five percent margin of error, the Raosoft sample size calculator calculated a sample size of 402 from the total population of the Hail city which is estimated at 731,000. The questionnaire includes demographic characteristics (i.e. age, gender, marital status, etc.) as well as a 7-item questionnaire to measure the awareness of the DM population regarding CKD. The survey was shared via various social platforms. A *p* value less than 0.05 is considered significant. To present the findings, tables and graphs are used. The study's contribution is to determine the level of awareness of the chronic renal disease among diabetes patients at the community level in the Hail region, Saudi Arabia, in 2022.

## 3. Statistical Analysis

The calculation of the awareness total score was drawn from 7-item questionnaires with “yes” coded as 1 and “no/I do not know” coded as 0 were the answer options. The overall score has been obtained by combining all 7 items. A possible score range from 0 to 7 has been generated, which indicates that the higher the score the higher the awareness of CKD. By using 50% and 75% as cutoff points to determine the level of awareness, participants were organized as having poor awareness if the score was from 0 to 3 points, 4 to 5 were considered moderate awareness, and 6 to 7 were considered as good awareness level.

The article "Measuring the Awareness of Chronic Kidney Disease (CKD) with Environmental Evaluation among Adult Diabetic Patients in Hail Region, Saudi Arabia" was retracted in 2023. Reasons: unreliable results or conclusions; concerns about the data; concerns about the peer review; concerns about the citations.

Measures of central tendency and dispersion were used to analyze the continuous (numerical) variables. All the categorical (nominal) data were presented as numbers and percentages. The comparison between the score of awareness and the demographic characteristics of the patients had been conducted using the Mann–Whitney *Z*-test as well as the Kruskal–Wallis *H*-test. Two-tailed analysis with *p* < 0.05 was used as a cutoff for statistical significance. The normality test was performed using the Shapiro–Wilk test. All data analyses were performed using the Statistical Package for Social Sciences, version 26 (SPSS, Armonk, NY : IBM Corp, USA).

## 4. Results

A total of 400 diabetic patients were recruited. As described in Table 1, the commonest age group was more than 40 years old (37%) with more than half (51%) being females. With regards to education, nearly 60% were bachelor's degrees. Married patients constitute 52.3% and 38% were employed. Patients with type 2 diabetes were reported by 23.8% and 40.5% had a DM duration of 5–15 years.

Figure 1 depicted patients' sources of CKD information. It can be observed that the most common source of information was the doctor (44.5%), followed by the Internet (22.5%), and friends and relatives (20.3%).

Table 2 shows the assessment of awareness of CKD among diabetic patients. Following the results, it can be shown that 63.7% of the patients knew that diabetes is a major cause of CKD, and 48.8% believed that all diabetics should have a periodic kidney function analysis. The proportion of the patients who believed that there are effective ways to avoid CKD was 54.8% while the proportion of patients who knew the symptoms associated with CKD was 45% and those who were aware of the complication of CKD was 43.5%. Patients who believed that early screening and treatment of CKD can reduce the risk of kidney failure were 62.7%. Finally, 53.% of the patients underwent a kidney function test. The overall awareness score was 3.71 (SD 2.14).

In Figure 2, the level of knowledge toward CKD among diabetic patients was poor, moderate, and good among 46.8%, 29.2%, and 24%, respectively.

The article "Measuring the Awareness of Chronic Kidney Disease (CKD) with Environmental Evaluation among Adult Diabetic Patients in Hail Region, Saudi Arabia" was retracted in 2023. Reasons: unreliable results or conclusions; concerns about the data; concerns about the peer review; concerns about the citations.

When measuring the association between the awareness score and the sociodemographic characteristics of the patients, it was observed that a higher awareness score was more associated with being a bachelor's degree (*Z* = 3.201; *p*=0.001), being unmarried (*Z* = 2.883; *p*=0.004), being a student (*H* = 22.651; *p* < 0.001), and having a doctor as a source of CKD information (*H* = 62.208; *p* < 0.001). Other variables showed no significant association with awareness score including age group, gender, type of diabetes, and duration of diabetes (*p* > 0.05) (see Table 3).

## 5. Discussion

The goal of this study was to determine the level of awareness of the chronic renal disease among diabetes patients. Our results showed that the awareness level of the patients regarding CKD was low. 46.8% of the patients appeared to have poor awareness levels, 29.2% were moderate and only 24% were shown to have a good understanding of the disease. Several studies established a low level of awareness in patients and their caregivers [1, 7, 15–20]. However, in Palestine [19], hypertensive individuals scored higher on total knowledge and attitude toward chronic renal disease prevention and early detection. The study further highlights the importance of having good knowledge, as well as a good attitude toward CKD, as improving both dimensions, had a relatively good chance of preventing CKD and its progression.

Education came out as a significant factor of awareness, where patients with bachelor's degrees exhibited better awareness levels than patients who are less educated. This is consistent with the report of Sa'adeh et al. [19], as well as Ahmed et al. [21], who reported that greater knowledge levels were significantly predicted among patients with higher educational levels. However, this has been contradicted by the report of Plantinga et al. [20]. After controlling for other variables, they discovered that wealth and educational levels had no effect on awareness of the personal risk of CKD status. They also stated that additional social factors such as marital status, social support, and having friends or acquaintances with CKD have yet to be investigated more in relation to CKD awareness. However, in our study, we managed to find a significant association between marital status and the level of awareness of patients about CKD, suggesting that unmarried patients tend to be more aware of CKD than married patients. More investigations are required in order to establish the true effect of social status on the CKD awareness level. Additionally, we noted that being a student likely to demonstrate a better understanding of the disease compared to other DM patients which may also need further investigations.

The article "Measuring the Awareness of Chronic Kidney Disease (CKD) with Environmental Evaluation among Adult Diabetic Patients in Hail Region, Saudi Arabia" was retracted in 2023. Reasons: unreliable results or conclusions; concerns about the data; concerns about the peer review; concerns about the citations.

In Palestine [19], a study found that patients who were less than 65 years were associated with higher knowledge scores of the disease. However, a study published in the USA [20], saw age as unrelated to the awareness level but they hypothesized that men with CKD would be more aware of their disease condition than women. In our study, both gender and age did not differ significantly with the level of awareness which did not coincide with previous results.

Our patients usually obtained CKD information from the doctor (44.5%), and it showed significant relation with awareness. Other sources of CKD information were the Internet (22.5%) and friends and relatives (20.3%). The source of information is one of the best ways to improve awareness. Our patients were shown to have the best source of the disease which is the ‘doctor.' In Jeddah, Saudi Arabia [22, 23], respondents preferred campaigns as a way to increase their awareness (59%) followed by media (48.5%). They further added that high-income participants were more likely to select clinics, campaigns, and the media as the best sources of CKD information.

The lack of awareness of CKD in our patients stemmed from the specific assessment of their understanding of the disease. For instance, poor awareness was shown about the complication of CKD (43.5%), as well as symptoms associated with CKD (45%). More than half of them (51.2%) were against the opinion that all diabetic patients should undergo a regular kidney function test even if asymptomatic. On the other hand, a handful of patients were knowledgeable that DM is a major cause of CKD (63.7%) and were aware that early screening and treatment can reduce the risk of kidney failure (62.7%). Conversely, patients were shown modest knowledge about the effective ways to avoid CKD (54.8%) and undergoing kidney function tests (53%). Consistent with our findings, a study conducted in Al Ahsa governorate showed that 52.8% of participants were aware that diabetes can lead to CKD, only 26.9% were unaware of the link between CKD and uncontrolled DM, and only 20.4% had never heard of CKD. However, a deficiency in the knowledge about the effective ways to prevent CKD (50%), the worst complication of CKD (29.3%), and the knowledge to notice the symptoms of CKD (14.5%) were shown in patients with diabetes [16, 24]. It is widely agreed that public awareness initiatives are required to enhance public awareness of CKD, its progression, and its complications.

## 6. Conclusion

Diabetic patients in our region are lacking awareness. Patients who were single with better education and who were well informed by the doctors about CKD information tend to be more aware of CKD as compared to other DM patients. The awareness levels among DM patients must be improved to prevent CKD, its development, and its complications. More efforts are needed to address the lack of awareness among diabetic patients. This can be done through awareness dissemination of CKD basic information. Further research is warranted in order to establish the awareness level of DM patients regarding CKD and its complications.

The article "Measuring the Awareness of Chronic Kidney Disease (CKD) with Environmental Evaluation among Adult Diabetic Patients in Hail Region, Saudi Arabia" was retracted in 2023. Reasons: unreliable results or conclusions; concerns about the data; concerns about the peer review; concerns about the citations.

## Figures and Tables

**Figure 1:** Sources of CKD information.

**Figure 2:** Level of awareness toward CKD.

**Table 1:** Demographic characteristics of the diabetic patients (*n* = 400).

Study data	*N* (%)
Age group	
18–20 years	54 (13.5%)
21–30 years	135 (33.8%)
31–40 years	63 (15.8%)
>40 years	148 (37.0%)

Gender	
Male	196 (49.0%)
Female	204 (51.0%)

Educational level	
Illiterate	23 (05.8%)
Primary school	14 (03.5%)
Elementary school	31 (07.8%)
High school	97 (24.3%)
Bachelor degree	235 (58.8%)

Marital status	
Single	170 (42.5%)
Married	209 (52.3%)
Divorced	21 (05.3%)

Occupation	
Student	125 (31.3%)
Employed	152 (38.0%)
Unemployed	123 (30.8%)

Type of diabetes	
Type 1	70 (17.5%)
Type 2	95 (23.8%)
I do not know	235 (58.8%)

Duration of diabetes	
<5 years	137 (34.3%)
5–15 years	162 (40.5%)
>15 years	101 (25.3%)

**Table 2:** Assessment of awareness of chronic kidney disease (CKD) among diabetic patients (*n* = 400).

Awareness statement	Yes (%)
1. Did you know that diabetes is a major cause of chronic kidney disease?	255 (63.7%)
2. Do you think that all diabetics should do a periodic kidney function analysis even if they were asymptomatic?	195 (48.8%)
3. Do you believe that there are efficient ways to avoid chronic kidney disease?	219 (54.8%)
4. Are you aware of any of the symptoms associated with chronic kidney disease?	180 (45.0%)
5. Are you aware of the complications of chronic kidney disease?	174 (43.5%)
6. Early screening and treatment of chronic kidney disease can reduce the risk of kidney failure?	251 (62.7%)
7. Have you ever done a kidney function test?	212 (53.0%)
Total awareness score (mean ± SD)	3.71 ± 2.14

**Table 3:** Association between the awareness and the sociodemographic characteristics of the diabetic patients (*n* = 400).

Factor	Awareness Score (7) Mean ± SD	*Z*/*H*-test	*p* value
Age group^a^			
≤30 years	3.93 ± 2.18	*Z* = 1.804	0.071
>30 years	3.53 ± 2.10		

Gender^a^			
Male	3.88 ± 2.10	*Z* = 1.534	0.125
Female	3.55 ± 2.18		

Educational level^a^			
High school or below	3.32 ± 2.10	*Z* = 3.201	0.001^*∗∗*^
Bachelor degree	3.99 ± 2.13		

Marital status^a^			
Unmarried	4.05 ± 2.06	*Z* = 2.883	0.004 ^*∗∗*^
Married	3.41 ± 2.18		

Occupation^b^			
Student	4.34 ± 2.07	*H* = 22.651	<0.001^*∗∗*^
Employed	3.75 ± 2.17		
Unemployed	3.03 ± 1.99		

Type of diabetes ^*∗*^^a^			
Type 1	3.93 ± 1.93	*Z* = 1.084	0.279
Type 2	3.62 ± 2.21		

Duration of diabetes^b^			
<5 years	3.36 ± 2.11	*H* = 5.951	0.051
5–15 years	3.83 ± 2.02		
>15 years	4.01 ± 2.33		

Source of CKD information^b^			
Doctor	4.62 ± 2.05	*H* = 62.208	<0.001^*∗∗*^
Friends and relatives	2.69 ± 1.81		
Internet	3.44 ± 1.96		
Others	2.67 ± 1.96		

^*∗*^Patients who did not know their diabetes type were excluded from the analysis. ^a^*p* value has been analyzed using the Mann–Whitney *Z*-test. ^b^*p* value has been analyzed using the Kruskal–Wallis *H*-test. ^*∗∗*^Significant at *p* < 0.05level.

The article "Measuring the Awareness of Chronic Kidney Disease (CKD) with Environmental Evaluation among Adult Diabetic Patients in Hail Region, Saudi Arabia" was retracted in 2023. Reasons: unreliable results or conclusions; concerns about the data; concerns about the peer review; concerns about the citations.

## Data Availability

The data used to support the findings of this study are included within the article.
